# Endothelial Cell Markers in Patients with Pseudoexfoliation Syndrome

**DOI:** 10.1100/2012/863949

**Published:** 2012-04-19

**Authors:** Joanna Stafiej, Grażyna Malukiewicz, Hanna Lesiewska-Junk, Danuta Rość, Karolina Kaźmierczak

**Affiliations:** ^1^Department of Ophthalmology, Ludwik Rydygier's Collegium Medicum, The Nicolaus Copernicus University, Curie-Skłodowskiej 9, 85-094 Bydgoszcz, Poland; ^2^Department of Pathophysiology, Ludwik Rydygier's Collegium Medicum, The Nicolaus Copernicus University, Curie-Skłodowskiej 9, 85-094 Bydgoszcz, Poland

## Abstract

The aim of the study was the assessment of the von Willebrand antigen (vWF Ag), E-selectin, and P-selectin concentration in blood plasma of patients with pseudoexfoliation syndrome (PEX). The group studied comprised 30 patients with PEX, aged from 50 to 86 years (mean 73, SD ± 8 years). Patients with cardiovascular and cerebrovascular diseases, diabetes mellitus, infectious disease, cancer, renal or liver insufficiency, connective tissue disease, current smoking, and hormone, antiplatelet, hypolipidemic, antioxidant, or antihypertensive drug therapy were excluded from the study. Each subject underwent a complete ophthalmological examination. Venous blood samples from the cubital vein were taken into sodium citrate solution. VWF Ag, sP-selectin, and sE-selectin concentration were determined by a commercially available enzyme-linked immunosorbent assay (MedSystems, Diagnostica Stago/Roche, R&D). Concentrations of vWF Ag, soluble E-selectin, and soluble P-selectin in blood plasma in the study group were compared with the levels in blood plasma in the control group. No significant differences were found between the groups. Our results indicate that there might be no correlation between PEX and such endothelial cell markers as vWF Ag, sP-selectin, and sE-selectin concentrations. Since the study size is limited, further investigations to confirm that there is no association between endothelial dysfunction in PEX and risk of future cardiovascular disease are necessary.

## 1. Introduction

Pseudoexfoliation syndrome (PEX) is a common age-related fibrillinopathy of unknown cause, primarily manifested in eyes by the accumulation of microscopic granular amyloid-like protein fibers. Originally, PEX was thought to be limited to the anterior segment of the eye, recent studies have indicated, however, that pseudoexfoliative material may be present in blood vessels; impaired endothelial function can be observed [1–3]. Since endothelial dysfunction is an independent predictor of future cardiovascular events, its presence in PEX syndrome patients might suggest an increased vascular risk [4–6]. Connection between inflammatory markers and markers of endothelial dysfunction favours the hypothesis that also inflammation could be involved in the etiopathogenesis of vascular disease [7]. An established marker of endothelial damage or dysfunction is von Willebrand factor (vWF) which is considered as biomarker in etiologic pathway of arteriosclerotic vascular disease [8]. The selectin family of cellular adhesion molecules (CAMs) plays a prominent role in immune/inflammatory responses [9, 10]. The aim of our study is to determine concentrations of biomarkers which may, according to the literature [11], precede the symptoms of vascular diseases, in patients with PEX and no other ocular nor systemic diseases. The present study is, to the best of our knowledge, the first one to evaluate vWF Ag and sCAMs levels in serum of patients with pseudoexfoliation syndrome.

## 2. Patients and Methods

Among 143, consecutive patients with PEX 113 were excluded based on general or ocular exclusion criteria. This prospective study involved 30 patients (18 females and 12 males) and 37 control subjects (25 females and 12 males) without PEX nor any history of systemic disease.

The study has been approved by the Medical Ethics Committee of Collegium Medicum Bydgoszcz Nicolaus Copernicus University in Toruń. Written informed consent was obtained from all study participants. A detailed medical history was collected from all subjects. Patients with cardiovascular diseases (defined as a history of myocardial infarction, angina pectoris, heart failure, left ventricular dysfunction, and peripheral arterial disease), diabetes mellitus, hypertension, cerebrovascular disease, infectious disease, cancer, renal or liver insufficiency, connective tissue disease, Parkinson's disease, current smoking, and hormone, antiplatelet, hypolipidemic, antioxidant or antihypertensive drug therapy were excluded from the study. Ocular exclusion criteria included a history of other than glaucoma neuropathies, anterior or posterior segment inflammation, chorioretinal degeneration, and retinal vascular diseases.

Each subject underwent a complete ophthalmological examination including slit lamp biomicroscopy after pupil dilation. Venous blood samples from the cubital vein were taken into sodium citrate solution (9 : 1). All venepunctures were performed using minimal venostasis, after 15 min in the recumbent position. In order to obtain low-platelet plasma, the blood samples were centrifuged at +4°C for 20 minutes with the speed of 3000 rotations per minute. The citrate plasma obtained in the procedure was divided into portions (approx. 200 *μ*L) placed in Eppendorf tubes. The material was then frozen in the temperature of −70°C until the study was being conducted. Von WF concentration, E-selectin and P-selectin levels were determined by a commercially available enzyme-linked immunosorbent assay using kits produced by Bender MedSystems, Diagnostica Stago/Roche, R&D.

**Statistical Analysis**

The Mann Whitney *U* test was used to compare patient and control groups for possible differences in vWF concentration and E-selectin and P-selectin levels.

## 3. Results

 The group studied comprised of 60% women and 40% men and similar rate was observed in the control one (68% versus 32%). There was no significant difference between study and control group in regards of gender.

Mean age in the studied group was 73 years (SD = 8) and in control one −57 (SD = 10).

The level of vWF Ag was not markedly elevated in patients with PEX, as compared to the controls (*P* = 0.5748). No significant differences were found in sE-selectin (*P* = 0.9666) and sP-selectin (*P* = 0.0519) levels between the patients with PEX syndrome and the control group. Detailed results are presented in Table 1.

## 4. Discussion

The etiology and pathophysiology of PEX still remain unexplained. Increased prevalence of the disease in certain populations and observed familial aggregation are compatible with PEX being a complex genetic disorder. A strong association between two nonsynonymous single nucleotide polymorphisms (SNPs) in the LOXL1 gene and PEX was detected [12–16]. Lysyl oxidase (LOX) belongs to a family of extracellular copper-requiring enzymes that facilitate cross-linking of collagen and elastane through oxidative deamination of lysine or hydroxylysine side chains and play a key role in collagen and elastane stabilizing. For over 10 years, PEX has been considered a systemic disease. There are also suggestions that this disease is linked to disorders impairing blood vessels [2]. Many authors have observed a connection between pseudoexfoliation syndrome and cardiovascular or cerebrovascular diseases [4, 11, 17–19]. Yet, there are no reports concerning the difference between PEX which is accompanied with other morbidities and that without such comorbidities.

Allingham et al. indicated in their study that pseudoexfoliation syndrome was strongly associated with the presence of glaucoma, but was associated with neither AMD nor systemic diseases [20].

Biomarkers of endothelial injury such as vWF, E-selectin, and P-selectin have been implicated in the development and progression of vascular diseases [7, 11, 21–27]. So far there are no reports on correlation between LOXL1 activation and endothelial dysfunction, vascular injury nor vWF/selectins. Elevated levels of vWF, sE-selectin, and sPselectin may develop as a result of endothelial damage mediated by hypertension. That's why patients displaying such diseases were excluded from the study. The lack of statistically significant differences in vWF Ag, sE-selectin, and sP-selectin levels between the group of PEX patients and the control group in our study suggests that there is no correlation between PEX and endothelial dysfunction. Thus, nonincreased level of the selectins in patients with PEX may indicate the lack of connection between this syndrome and vascular diseases. Other authors' results also support such a conclusion [28–30]. However, it is possible that other factors, such as thrombogenicity, are enhanced in PEX and this would increase the risk of cardiovascular event. Although PEX is thought to be related with cardiovascular diseases, our research casts doubt on the existence of such a link. Similarly, Tarkkanen in his review concluded that there is no evidence that pseudoexfoliation syndrome or pseudoexfoliation glaucoma are related to increased mortality from cardiovascular diseases [31]. Nevertheless, the underlying pathogenesis of PEX might be multifactorial. Because hitherto, a clearcut association of PEX with asystemic diseases is yet to be shown, further large-scale, randomized clinical studies are required.

## 5. Conclusion

Our results indicate that there might be no correlation between PEX and vWF Ag, sP-selectin, and sE-selectin endothelial cell markers concentrations. The study size is limited therefore further investigations are required to confirm the lack of association between endothelial dysfunction and PEX.

## Figures and Tables

**Table 1:** Endothelial cell markers in blood plasma of patients with PEX and controls.

Parameter	Study group (median, Quartile1 & Quartile3)	Control group (median, quartile1, quartile3)
von Willebrandt antigen (%)	67,77 Q1 = 53,59 Q3 = 80,89	66,36 Q1 = 59,55 Q3 = 81,82

sE-selectin (ng/mL)	40,27 Q1 = 27,94 Q3 = 54,64	40,94 Q1 = 33,16 Q3 = 60,12

sP-selectin (ng/mL)	86,85 Q1 = 71,16 Q3 = 110,72	100,97 Q1 = 70,35 Q3 = 146,19
